# Warning and Nursing Experience of Anesthesia Depth Monitoring for Patients with General Anesthesia Delayed to Leave Anesthesia Recovery Room and Delirium

**DOI:** 10.1155/2022/3610838

**Published:** 2022-11-10

**Authors:** Hongmei Xuan, Keping Xu

**Affiliations:** ^1^Department of Pain, Zhuji People's Hospital of Zhejiang Province, Zhuji, Shaoxing 311800, Zhejiang, China; ^2^Department of Anesthesia, Zhuji Traditional Chinese Medicine Hospital of Zhejiang Province, Zhuji, Shaoxing 311800, Zhejiang, China

## Abstract

Affected by the residues of narcotic drugs, patients under general anesthesia are vulnerable to emergence of agitation, delirium, hemodynamic changes, and other adverse events in the recovery period of anesthesia. Therefore, it is necessary to strengthen the observation and care of these patients. Depth of anesthesia monitoring (DAM) has always been a concern for anesthesiologists, but there are few reports related to it. This study compared the early warning value of DAM for patients under general anesthesia with delayed exit from the anesthesia recovery unit (PACU) and delirium and summarized the related nursing experience. The results showed that DAM could reduce the incidence of complications in patients under general anesthesia, reduce the incidence of delirium, shorten the time of postoperative anesthesia recovery and PACU observation time, reduce the workload of nursing staff, and improve nursing satisfaction. DAM plays an important role in improving the quality and efficiency of care in PACU.

## 1. Introduction

General anesthesia is the key to ensure the smooth progress of surgery. However, since the functions of various tissues and organs of the patient's body are in an unstable state during the anesthesia recovery period after general anesthesia, and it is difficult to accurately control the dose of clinical anesthetics, anesthetic residues often appear in the recovery process, which may cause delirium, low oxygen saturation, nausea and vomiting, aspiration, and hypotension, and affect the surgical efficacy [1, 2]. Postanesthesia care unit (PACU) is mainly used for condition change monitoring and treatment recovery after surgical anesthesia and before the patient's vital signs are unstable [3]. All patients need to be transferred to PACU after surgery until recovery, so PACU nursing work plays an important role in postoperative recovery and safety of anesthetized patients. Relevant studies have shown that depth of anesthesia monitoring (DAM) can help medical staff to grasp the depth of anesthesia in a timely manner, conduct reasonable interventions in a timely manner, and ensure the safety of patients to the greatest extent [4]. However, there are few reports related to the effect of deep anesthesia monitoring on patients under general anesthesia. Based on this, the author compares the effects of DAM technology on delayed out of PACU, occurrence of delirium, and nursing work in this study. The report is as follows.

## 2. Materials and Methods

### 2.1. Research Objects

100 patients who underwent general anesthesia in our hospital from January 2019 to January 2020 were selected, including 32 males and 18 females in the control group. The patients were divided into the experimental group (*n* = 50) and the control group (*n* = 50) according to the random number method. This study was approved by the Medical Ethics Committee.

### 2.2. Inclusion Criteria

The inclusion criteria are as follows: (1) patients meeting the indications for general anesthesia [5]; (2) patients whose operation time exceeds two hours; (3) patients whose American Association for Standardization (ASA) anesthesia classification [6] is between grade II and III; (4) patients whose body mass index (BMI) ≤ 30 kg/m^2^; and (5) patients who have signed informed consent form.

### 2.3. Exclusion Criteria

Exclusion criteria are as follows: (1) patients with contraindications to surgery; (2) patients with allergies to anesthetics; (3) patients with severe insufficiency of organs such as the heart, liver, kidney, or lung; (4) patients with preoperative disturbance of consciousness or mental illness; and (5) general information is incomplete or the researcher quits midway.

### 2.4. Treatment Methods

The patients in both groups received general anesthesia with tracheal intubation, and after entering the operating room, they were given open venous channel and continuous intravenous infusion of 500 ml compound sodium chloride injection. Oxygen was inhaled through nasal catheter, and the oxygen flow was set at 3-5 L/min. Patients were monitored by routine ECG monitoring such as respiration, blood pressure, pulse, oxygen saturation, and ECG. After entering the operating room, the anesthesiologist made appropriate adjustments to the infusion rate and dose of anesthetic drugs according to the specific situation during the operation.

On this basis, the patients in the test group were connected with BIS VISTA monitor (Aspect Medical Systems, Inc) after entering the operating room. The bispectral index (BIS value) of electroencephalogram was detected, and the depth of anesthesia was adjusted according to the BIS value. The value was maintained at 50-60, and the two groups of patients were sent to PACU for observation. Anesthesia was induced with propofol, sufentanil, and cisatracurium. After the operation, in the operating room, the respiratory rate of the two groups was more than 12 times/min and SPO_2_ extubation can be performed if the tidal volume exceeds 95% and the tidal volume reaches 6 ml/kg.

### 2.5. Observation Indicators and Evaluation Criteria

1. Compare the dose of anesthesia between the two groups.
2. Vital signs in different time periods: the mean arterial pressure (MAP), heart rate (HR), and SPO_2_ at the beginning of surgery (T0), extubation (T1), 10 minutes after extubation (T2), and the time to leave the PACU (T3) were compared between the two groups.
3. Compare the extubation time between the two groups.
4. Compare the PACU observation time between the two groups.
5. Delirium assessment: professional training is provided to the investigator before the study, and the delirium is scored by the investigator after the patient wakes up and is extubated. The simplified Chinese version of Nu-DESC (Nu-DESC-SCV) was used to evaluate the delirium degree of patients in two groups. Five items were scored from delusions\hallucinations, disorientation, abnormal behavior, abnormal verbal communication, and psychomotor retardation. Score is given according to the severity of the patient: 0 is absent, 1 is mild, and 2 is moderate to severe [7].
6. Compare the nursing satisfaction between the two groups.
7. Nursing activity assessment scale (NAS) [8]: it consists of 23 nursing items from 5 aspects, including activities, testing, health care, nursing administration, and patient support for nursing work. The higher value indicates greater workload. As a nursing quality evaluation standard, each item corresponds to a score of 1.2-32.0 according to the percentage of nurses' 24-hour working time. The higher score is, the greater the workload. The patient's 24 h NAS score ranges from 0 to 177 points, working hours = score/100*∗*24 h, starting from the patient's end of surgery and entering the PACU for resuscitation, until leaving the PACU and returning to the ward.
8. Compare the incidence of complications between the two groups.

### 2.6. Statistical Methods

All data were processed by SPSS23.0 statistical software package. The continuous variable data of experimental data were expressed as mean standard deviation ($\bar{x}$ ± *s*) and adopted *t*-test. The classified variable data and descriptive analysis were expressed as (%) and adopted *χ*^2^ test. *P* < 0.05 was considered statistically significant.

## 3. Results

### 3.1. General Data

There was no significant difference in the general data between the two groups (*P* > 0.05), and they were comparable. See Table 1 for details.

### 3.2. Comparison of the Dose of Anesthesia, Extubation Time, and Observation Time between the Two Groups

The doses of propofol and cisatracurium used in the test group were less than those in the control group (*P* < 0.05), but the doses of sufentanil used in the two groups were not statistically significant (*P* > 0.05). The extubation time and observation time were longer than those in the experimental group (*P* < 0.05). See Table 2 for details.

### 3.3. Comparison of Vital Signs between Two Groups of Patients at Different Time Periods

The MAP and HR in the T1 and T2 time periods of the two groups were higher than those in T0 (*P*< 0.05), and the MAP and HR in the T1 and T2 time periods of the experimental group were higher than those of the control group (*P* < 0.05). There was no difference in SPO_2_ level between the two groups at any time point (*P* > 0.05). See Table 3 for details.

### 3.4. Comparison of Delirium Assessment and Complications between Two Groups of Patients

The Nu-DESC-SCV score of the experimental group was significantly lower than that of the control group (*P* < 0.05). See Table 4 for details.

### 3.5. Comparison of Nursing Satisfaction and Nursing Quality Assessment between the Two Groups

The NAS score of the test group was lower than that of the control group, and the nursing satisfaction degree was higher than that of the control group (*P* < 0.05). See Table 5 for details.

### 3.6. Comparison of Complications between the Two Groups

The incidence of complications in the experimental group and the control group were 14% and 32%, respectively. The incidence of complications in the experimental group was lower than that in the control group (*P* < 0.05). See Table 6 for details.

## 4. Discussions

The functions of various systems and organs of the body are in an unstable state for a period of time after the operation under general anesthesia [9]. At the same time, because of the residual effects of anesthetics and muscle relaxants and the failure to normalize protective reflexes, a series of adverse events, including postoperative delirium, often occur. Delirium can cause disorders of consciousness, memory, perception, and even other organ functions. Besides, the death rate caused by delirium is relatively high, and research results show that the death rate ranges from 22% to 76% [10]. Therefore, avoiding the occurrence of delirium after general anesthesia is of great significance to the prognosis of patients.

In this study, the doses of propofol and atracurium used in the experimental group were lower than those in the control group (*P* < 0.05), suggesting that DAM could save anesthetics and avoid excessive anesthesia. At the same time, the incidence of respiratory complications, consciousness disorders, nausea, and vomiting complications in the experimental group was significantly lower than that in the control group (*P* < 0.05), indicating that DAM can effectively improve the quality of patients' rehabilitation, reduce the incidence of complications, and improve the perioperative outcome. The possible reason for the above results is that in the past, the traditional depth of anesthesia was determined based on the changes in patients' heart rate and blood pressure level [11]. However, under the influence of factors such as surgical invasive operations during the operation, it may lead to the increase of reflex sexual intercourse sensation activity of the body, which will gradually become stable after a period of time. At this time, the judgment of the depth of anesthesia may be affected, further affecting the postoperative anesthesia recovery. However, DAM results allow for the development of individualized anesthesia regimens that assure the reasonableness of sedative doses [12]. This effectively ensures the rationality of the anesthesia depth, prevents the awareness during the operation and excessive stress response of the body caused by the insufficient anesthesia depth, thereby reducing the occurrence of perioperative adverse events, and also effectively reduces the exposure of anesthetics in the operation of patients, thereby shortening the awakening time and respiratory function recovery time after the operation [13, 14].

The mechanism of postoperative delirium has not been clearly explained, but most scholars believe that it may be related to neuronal differentiation ability, cognitive reserve, cerebral blood flow, cognitive function, decreased brain volume, and large fluctuations in endocrine levels, which may lead to patients' tolerance to anesthesia force drop related [15, 16]. Therefore, in anesthesia monitoring, a method that has little impact on the body, less interference with physiological functions, and effectively inhibits surgical stimulation energy should be selected. Nu-DESC-SCV is a rapid, easy-to-use, and convenient nursing delirium screening scale [17]. In this study, the MAP and HR of the experimental group during T1 and T2 were higher than those of the control group, and the Nu-DESC-SCV score of the experimental group was significantly lower than that of the control group (*P* < 0.05), indicating that DAM can effectively reduce the incidence of delirium and improve vital signs in patients. This may be related to the accurate regulation and judgment of the depth of anesthesia by DAM, avoiding the stress response or EEG burst suppression caused by the discomfort of deep and shallow anesthesia, and reducing the exposure of anesthetics [18, 19]. PACU care is an important part of this. Studies have shown that the NAS score of some hospitals is 68.64, which indicates that nursing staff are in a state of full load or even overload in most cases [20]. In this study, the NAS score of the control group was higher than that of the experimental group, and the nursing satisfaction was lower than that of the experimental group (*P* < 0.05). This shows that DAM can significantly improve work efficiency, reduce PACU nursing workload, and improve nursing quality. The reason is that DAM can effectively shorten the awakening time, reduce observation time, improve vital signs and reduce the incidence of complications, to a certain extent, and reduce the workload of nursing care, which makes the nursing work more efficient.

In conclusion, DAM can reduce the incidence of complications in patients with general anesthesia, reduce the incidence of delirium, shorten postoperative anesthesia recovery time and PACU observation time, reduce the workload of nursing staff, improve nursing satisfaction, improve the quality of PACU nursing work and efficiency. However, the shortcomings of this study lie in the fact that the included sample size is small and too centralized. Further prospective multicenter research is needed to investigate the effects and related mechanisms of DAM in patients undergoing surgical anesthesia from different regions, different levels of hospitals, and different populations.

## Figures and Tables

**Table 1:** Comparison of general information of patients (n (%), $\bar{x}$ ± *s*).

Group	*n*	Age (year)	Gender		Weight (kg)	ASA stage			Operation time (h)
			Male	Female		I	II	III	
Control group	50	51.62 ± 10.10	32	18	49.15 ± 7.12	20	26	4	2.51 ± 0.24
Test group	50	52.15 ± 9.23	30	20	50.45 ± 7.54	19	28	3	2.43 ± 0.32
*t/χ * ^2^ value	—	0.274	0.170	0.886			0.243		1.412
*P*-value	—	0.785	0.680	0.378			0.886		0.161

**Table 2:** Comparison of anesthesia dose, extubation time, and observation time between two groups of patients ($\bar{x}$ ± *s*).

Group	*n*	Propofol (mg)	Sufentanil (ug)	Cisatracurium (mg)	Extubation time (min)	Observation time (min)
Control group	50	110.56 ± 23.35	12.36 ± 3.36	13.34 ± 4.32	8.74 ± 2.15	52.85 ± 10.65
Test group	50	102.24 ± 12.64	11.51 ± 2.31	9.64 ± 2.65	5.47 ± 1.52	30.12 ± 6.21
*t*-value	—	2.216	1.474	5.162	8.782	13.037
*P*-value	—	0.029	0.144	0.001	0.001	0.001

**Table 3:** Comparison of vital signs between two groups of patients at different time periods ($\bar{x}$ ± *s*).

Group	*n*	Time	MAP (mmHg)	HR (b/m)	SPO_2_ (%)
Control group	50	T0	82.65 ± 11.52	71.36 ± 14.62	98.64 ± 5.62
		T1	94.62 ± 16.35^a^	86.14 ± 13.52^a^	97.56 ± 4.72
		T2	86.15 ± 14.22^a^	77.12 ± 10.56^a^	95.41 ± 3.26
		T3	76.34 ± 10.54	71.25 ± 10.25	96.58 ± 5.36

Test group	50	T0	81.32 ± 10.24	72.24 ± 10.32	98.58 ± 5.63
		T1	97.24 ± 15.05^ab^	93.64 ± 16.67^ab^	96.47 ± 5.34
		T2	93.61 ± 14.36^ab^	85.47 ± 15.21^ab^	95.74 ± 4.34
		T3	80.54 ± 13.85	77.14 ± 13.25	97.14 ± 2.14

*Note.* Compared with T0, ^*a*^*P* < 0.05; compared with the control group at the same time, ^*b*^*P* < 0.05.

**Table 4:** Comparison of delirium assessment between the two groups ($\bar{x}$ ± *s*).

Group	*n*	Nu-DESC-SCV (score)
Control group	50	4.21 ± 1.35
Test group	50	2.12 ± 0.34
*t*-value	—	10.616
*P*-value	—	0.001

**Table 5:** Comparison of nursing satisfaction and nursing quality assessment between the two groups (n (%), $\bar{x}$ ± *s*).

Group	*n*	NAS (score)	Nursing satisfaction (%)
Control group	50	61.24 ± 9.64	38 (76.00)
Test group	50	57.56 ± 5.35	46 (92.00)
*t/χ * ^2^ value	—	2.360	5.314
*P*-value	—	0.020	<0.05

**Table 6:** Comparison of delirium assessment and complications between the two groups.

Group	Respiratory complication	Disturbance of consciousness	Sick/vomit	Complication rate
Control group (*n* = 50)	7 (14.00)	5 (10.00)	4 (8.00)	16 (32.00)
Test group (*n* = 50)	3 (6.00)	2 (4.00)	2 (4.00)	7 (14.00)
*χ * ^2^ value	—	—	—	4.574
*P*-value	—	—	—	0.032

## Data Availability

The data used and/or analyzed during the current study are available from the corresponding author.
